# Inhibition of inflammation using diacerein markedly improved renal function in endotoxemic acute kidney injured mice

**DOI:** 10.1186/s11658-018-0107-z

**Published:** 2018-08-16

**Authors:** Guangzhe Yu, Qian Liu, Xuening Dong, Kaihong Tang, Bohui Li, Chunmei Liu, Wenzheng Zhang, Yiduo Wang, Yingyu Jin

**Affiliations:** 1 Department of Emergency Surgery, The 1st Affiliated Hospital of Harbin Medical University, Harbin, Heilongjiang Province China; 2 Department of Laboratory Diagnosis, The 1st Affiliated Hospital of Harbin Medical University, 23 Youzheng Street, Nangang District, Harbin, 150001 Heilongjiang Province People’s Republic of China

**Keywords:** Endotoxemia, Acute kidney injury, Inflammation, Aquaporins, Sodium transporters, Diacerein

## Abstract

**Background:**

Inflammation is an important pathogenic component of endotoxemia-induced acute kidney injury (AKI), finally resulting in renal failure. Diacerein is an interleukin-1β (IL-1β) inhibitor used for osteoarthritis treatment by exerting anti-inflammatory effects. This study aims to investigate the effects of diacerein on endotoxemia-induced AKI.

**Methods:**

Male C57BL/6 mice were intraperitoneally injected with lipopolysaccharide (LPS, 10 mg/kg) for 24 h prior to diacerein treatment (15 mg/kg/day) for another 48 h. Mice were examined by histological, molecular and biochemical approaches.

**Results:**

LPS administration showed a time-dependent increase of IL-1β expression and secretion in kidney tissues. Diacerein treatment normalized urine volume and osmolarity, reduced blood urea nitrogen (BUN), fractional excretion of sodium (FENa), serum creatinine and osmolarity, and protected renal function in an endotoxemic AKI mice model. In the histopathologic study, diacerein also improved renal tubular damage such as necrosis of the tubular segment. Moreover, diacerein inhibited LPS-induced increase of inflammatory cytokines, such as IL-1β, tumor necrosis factor-α, monocyte chemoattractant protein-1 and nitric oxide synthase 2. In addition, LPS administration markedly decreased aquaporin 1 (AQP1), AQP2, AQP3, Na,K-ATPase α1, apical type 3 Na/H exchanger and Na-K-2Cl cotransporter expression in the kidney, which was reversed by diacerein treatment. We also found that diacerein or IL-1β inhibition prevented the secretion of inflammatory cytokines and the decrease of AQP and sodium transporter expression induced by LPS in HK-2 cells.

**Conclusion:**

Our study demonstrates for the first time that diacerein improves renal function efficiently in endotoxemic AKI mice by suppressing inflammation and altering tubular water and sodium handing. These results suggest that diacerein may be a novel therapeutic agent for the treatment of endotoxemic AKI.

## Background

Endotoxemia frequently occurs under extremely pathological stressful conditions, such as infection, burn, shock and trauma [1]. It plays a key role in the onset of acute injury of multiple organs, including acute kidney injury (AKI), which is characterized by a decreased glomerular filtration rate and rapid loss of renal function [2]. Lipopolysaccharide (LPS), a major constituent of gram-negative bacteria, is involved in the pathogenesis of endotoxemia-induced AKI [3].

Accumulating evidence has demonstrated that renal tubule function, including water reabsorption and urine concentration, is regulated by aquaporins (AQPs) and sodium transporters [4–6]. AQPs, a family of membrane proteins, play a critical role in regulating water balance [5]. A previous study reported that reduction of AQP expression was associated with renal tubular epithelial cell damage [7]. In contrast, elevation of AQP expression could improve water metabolism in the kidney, thereby relieving injury [5]. Moreover, it has been shown that endotoxemia decreased AQP2 expression, which is responsible for the decrease of urine osmolality [2]. In addition, the major fraction of sodium is reabsorbed at the kidney proximal tubule by Na,K-ATPase, apical type 3 Na/H exchanger (NHE3) and Na-K-2Cl cotransporter (NKCC2) [6]. During endotoxemia, proximal tubular cells, the primary target of endotoxemia, develop abnormal expression or distribution of sodium transporters, leading to impaired sodium reabsorption [8]. A marked decrease of Na,K-ATPase, NHE3 and NKCC2 has been observed in endotoxemic animals [4, 9], further indicating that dysregulation of sodium transporters may be closely related to abnormal proximal tubular sodium reabsorption. Therefore, modulation of AQP and sodium transporter expression may be a relevant therapeutic approach for endotoxemic AKI.

In addition to hemodynamic, metabolic, and systemic changes, inflammation has become a center of interest in kidney injury, along with increased levels of inflammatory cytokines, such as interleukin-1β (IL-1β), tumor necrosis factor-α (TNF-α) and monocyte chemoattractant protein-1 (MCP-1) [10, 11]. Inhibition of inflammation could attenuate the decrease of renal AQP and sodium transporter expression in rats with ischemia/reperfusion-induced AKI [12, 13]. Diacerein is an important IL-1β inhibitor, which has been approved as an oral anti-inflammatory agent for osteoarthritis treatment [14]. It is entirely converted into rhein by acetylation in the liver [15]. Multiple studies have demonstrated the anti-inflammatory ability of diacerein by inhibiting IL-1β synthesis and inflammatory cytokine production as well as IκB-α/NFκB pathway activation [16, 17]. Interestingly, recent studies have shown that diacerein could improve renal function in diabetic nephropathy in mice and obese insulin-resistant rats [18, 19], suggesting that diacerein may also play a protective role against kidney injury. Taking these aspects into consideration, we hypothesized in the present study that diacerein could ameliorate endotoxemia-induced kidney injury and dysfunction via inhibiting inflammation and maintaining AQP expression.

## Methods

### Animals

Eight-week old male wild-type C57BL/6 mice (20~ 25 g) were obtained from the Jackson Laboratory (CA, USA). The mice were bred and housed in cages with free access to water and diet at Harbin Medical University. To generate the endotoxemic AKI model, mice were injected intraperitoneally with 10 mg/kg LPS (100 μL) once and continued to 72 h. Diacerein (dissolved in DMSO, Sigma Aldrich, MO, USA) was injected intraperitoneally at a dose of 15 mg/kg (50 μL) and continuously dosed once a day for 2 days after 24 h of LPS challenge. All mice (*n* = 110) were randomly divided into 4 groups: control (*n* = 40), LPS (n = 40), LPS DMSO (*n* = 15), LPS Diacerein (n = 15). According to the time points (12, 24, 48 and 72 h), the first two groups were further divided into 4 subgroups (*n* = 10/group). No mice died during the experimental period.

### Quantitative real-time PCR

Total RNA from the mouse kidney tissues was isolated using the Qiagen RNeasy Kit (CA, USA) according to the manufacturer’s instructions. 2 μg of RNA was reverse-transcribed using the RevertAid First Strand cDNA Synthesis Kit (Thermo Fisher Scientific Inc., IL, USA). cDNA was mixed with the Fast SYBR Green Master Mix Kit (Applied Biosystems, CA, USA) and amplified using the 7500 Fast Real-Time PCR System (Applied Biosystems). Amplifications were carried out with the following cycling conditions: 95 °C for 10 min followed by 32 amplification cycles of denaturation (95 °C for 10 s), annealing (62 °C for 30 min) and extension (59 °C for 30 s). The IL-1β mRNA expression was normalized to the mRNA levels of GAPDH and calculated using the 2^-ΔΔCT^ method. The specific primer sequences used for the amplification were as follows: IL-1β, 5′-GTCAACGTGTGGGGGATGAA-3′ and 5′-AAGCAATGTGCTGGTGCTTC-3′; GAPDH, 5′-GGTTGTCTCCTGCGACTTCA-3′ and 5′-CCCTAGGCCCCTCCTGTTAT-3′.

### Histological analyses

Immunohistochemistry for IL-1β was performed on 5-μm paraffin-embedded slides from mouse kidney tissues in each group using the streptavidin-biotin-peroxidase complex system according to the supplier’s instructions (DAKO Japan, Tokyo, Japan). The slides were heated for 30 min at 65 °C, dewaxed in xylene, and rehydrated through graded ethanol at room temperature. The peroxidase was blocked by 5% H_2_O_2_ in methanol and non-specific staining was prevented by incubation with 1% bovine serum albumin (BSA). Slides were treated with IL-1β antibody (1:50) or F4/80 (1:100) (both from Santa Cruz Biotechnology, Santa Cruz, CA, USA) diluted in 0.1% BSA overnight at 4 °C. After rinsing with phosphate buffered saline (PBS) 3 times, the slides were incubated with biotinylated secondary antibody and developed by the streptavidin-peroxidase reaction using diaminobenzidine (DAB). For histopathological examination, the slides of kidney tissues were stained with hematoxylin and eosin (H&E). All slides were observed and examined under an Olympus light microscope (CKX41, Tokyo, Japan).

### Biochemical analysis

At the end of the experimental period, mice were placed in a metabolic cage at room temperature, allowing measurements of water intake and quantitative urine collections for 12 h. Animals were anesthetized with isoflurane, and a 28-gauge catheter was inserted into the right carotid artery for the determination of systemic mean arterial pressure (MAP) (model 66S; Hewlett Packard, Geneva, Switzerland). After measurement, blood samples were collected and centrifuged at 1200×g for 10 min at room temperature and the supernatant was transferred into sterile tubes for storage at − 80 °C. An automatic biochemical analyzer (Hitachi 7600, Hitachi, Tokyo, Japan) was used to determine blood urea nitrogen (BUN) and creatinine. Sodium concentration was tested using an IL 943 flame photometer (Instrumentation Labs, MA, USA) and fractional excretion of sodium (FENa) was calculated. Urine and serum osmolality were measured by freezing-point depression (Advanced Instruments, Norwood, MA, USA).

### Cell culture

The human renal proximal tubular epithelial HK-2 cell line was obtained from American Type Culture Collection (CRL-2190; VA, USA) and cultured in RPMI-1640 medium (Gibco BRL Life Technologies, CA, USA) supplemented with 0.5% heat-inactivated fetal bovine serum and 1% penicillin/streptomycin. In this study, the cells were pretreated with IL-1β siRNA for 48 h or diacerein (1 μM) for 1 h followed by LPS (1 μg/mL) incubation for another 48 h.

### Small interfering RNA experiments

The stealth siRNA targeting human IL-1β (5′-TGAACCTGTTCCAAAACTC-3′) and randomly scrambled siRNA (negative siRNA) were synthesized and purchased from Invitrogen (CA, USA). The HK-2 cells were transfected with 50 nM of IL-1β siRNA or negative siRNA using the RNAiMAX transfection reagent (Invitrogen) according to the manufacturer’s instructions. 48 h-interfered cells were subsequently incubated with LPS for a further 48 h at 37 °C.

### Enzyme-linked immunosorbent assay (ELISA)

Whole kidneys or HK-2 cells were homogenized in a buffer containing 250 mM sucrose, 1 mM EDTA, 25 mM imidazole, 0.1 mM phenylmethylsulfonyl fluoride (PMSF) and 20 mM potassium phosphate buffer (pH 7.6), with 1% protease and phosphatase inhibitors (Roche Applied Science, IN, USA) at 4 °C. Tissue samples were centrifuged at 10,000 g for 30 min at 4 °C. The supernatant was used for determination of inflammatory cytokine concentrations and western blotting. IL-1β, TNF-α, MCP-1 and NOS-2 were determined by a mouse IL-1β ELISA Kit, a TNF-α ELISA Kit, an MCP-1 ELISA Kit (Boster, Wuhan, China) and an NOS-2 ELISA Kit (Elabscience, CA, USA). Procedures were performed according to the manufacturer’s instructions.

### Western blotting

The protein concentration of kidney tissue samples or HK-2 cells was determined with the Enhanced BCA Protein Assay Kit (Beyotime, Shanghai, China). Equal amounts of protein (50 μg) were separated on 10% SDS-polyacrylamide gel electrophoresis and transferred to polyvinylidene fluoride (PVDF) membranes (Millipore, MA, USA), and were subsequently blocked by 5% non-fat milk powder in TBST (10 mM Tris-HCl, 150 mM NaCl, 0.05% Tween-20, pH 7.6) for 1 h. After blocking, membranes were incubated with primary antibodies against AQP1 (1:500), AQP2, Na,K-ATPase α1, NKCC2, NHE3, β-actin (1;1000) (Santa Cruz Biotechnology) and AQP3 (1:1000, Alomone Labs, Jerusalem, Israel). Then the membranes were washed with TBST and the primary antibodies were detected with horseradish peroxidase-conjugated secondary antibodies (Santa Cruz Biotechnology). The bands were visualized with enhanced chemiluminescence reagent (Pierce Biotech, IL, USA). Protein expression levels were determined by analyzing the signals captured on the membranes using the ImageJ software (NIH, Maryland, USA).

### Statistical analysis

Data were expressed as mean value ± standard error of mean (SEM) and compared by the two-tailed Student’s t test or one-way ANOVA, followed by the Bonferroni multiple comparison test. Statistical analysis was performed using SPSS 18.0 software (SPSS Inc., Chicago, IL, USA). *P* < 0.05 was considered statistically significant.

## Results

### Expression and secretion of IL-1β were elevated in endotoxemic AKI mice

Real-time PCR results showed that endotoxemia, induced by LPS, time-dependently increased renal IL-1β mRNA abundance. The mRNA expression of IL-1β was about 1.2-fold, 1.8-fold, 2.1-fold and 2.0-fold higher than that of control levels at 12 h, 24 h, 48 h and 72 h after LPS administration, respectively (Fig. 1a). ELISA results also indicated that LPS led to time-dependent induction of renal IL-1β secretion (Fig. 1b). Further, immunohistochemical studies demonstrated that the cytoplasmic immunoreactivity of IL-1β in the renal cortex and renal medulla was significantly increased in endotoxemic mice compared with control mice (Fig. 1c and d).

**Fig. 1:** LPS induced IL-1β level in mouse kidney tissues. **a** Interleukin-1β (IL-1β) mRNA expression was analyzed in kidney tissues from control or lipopolysaccharide (LPS)-treated mice by real-time PCR at the times as indicated. LPS time-dependently increased the IL-1β mRNA expression. **b** ELISA analysis showing time-dependent increase of renal concentrations of IL-1β after LPS treatment for 72 h compared with control group. **P < 0.01 vs. control, *n* = 8 in each group. **c** and **d** Immunohistochemical protein expression of IL-1β in renal cortex (**c**) and medulla (**d**) of mice after 72 h of LPS treatment (magnification, 200×). Arrows indicate the positive staining area of IL-1β

### Diacerein ameliorated renal injury in endotoxemic mice

To investigate whether IL-1β inhibitor diacerein protects against endotoxemic renal injury, mice were challenged with LPS followed by diacerein administration. Indicators of renal function were determined at the end of the experimental period. As displayed in Table 1, MAP did not differ between any of the four groups. LPS markedly decreased body weight compared with control mice, but it did not differ among LPS groups. Water intake, urine volume and osmolarity, and creatinine clearance were significantly decreased in LPS-treated mice, and were remarkably recovered by diacerein treatment. Moreover, diacerein also significantly inhibited the LPS-induced increase of serum creatinine, BUN, FENa and osmolarity. In addition to renal function, histological analysis was performed to confirm the protective effect of diacerein. In the cortex from LPS-treated mice, there was glomerular congestion and atrophy, interstitial hemorrhages, and epithelial cell necrosis and shedding (Fig. 2a). In the medulla, LPS also resulted in disruption of normal architecture, which was evidenced by erythrocyte extravasation, cast formation, tubular collapse and collecting duct necrosis (Fig. 2b). However, diacerein treatment clearly attenuated tubular damage induced by endotoxemia (Fig. 2).

**Table 1:** Hemodynamic and biochemical parameters

Parameter	Control	LPS		
		–	DMSO	Diacerein
Body weight (g)	21.4 ± 0.8	18.7 ± 1.0**	19.2 ± 0.9**	19.4 ± 0.4**
MAP, (mmg)	118.3 ± 12.4	102.4 ± 14.0	109.6 ± 11.8	114.1 ± 9.5
Water intake (ml/100 g/12 h)	5.8 ± 0.6	3.0 ± 0.4**	2.7 ± 0.5**	4.7 ± 0.3^##^
Urine volume (ml/100 g/12 h)	2.8 ± 0.5	1.0 ± 0.1**	1.2 ± 0.2**	2.2 ± 0.2^##^
Creatinine (mM)	22.1 ± 2.5	72.3 ± 2.8**	73.3 ± 5.1**	34.0 ± 2.1^##^
Creatinine clearance (mL/min/kg)	5.8 ± 0.3	3.9 ± 0.5**	4.2 ± 0.4**	5.3 ± 0.4^##^
BUN (mM)	5.6 ± 0.9	14.4 ± 1.1**	15.8 ± 1.5**	6.7 ± 0.8^##^
FENa (%)	0.6 ± 0.1	1.8 ± 0.3**	1.2 ± 0.1**	0.9 ± 0.2^##^
Urine osmolarity (mOsm/L)	3166 ± 192	1520 ± 84**	1487 ± 95**	2674 ± 114^##^
Serum osmolarity (mOsm/L)	314 ± 5	342 ± 3**	340 ± 6**	319 ± 2^##^

Variables were measured at the end of 72-h experimental period. Values are expressed as means±SEM, *MAP* mean arterial pressure, *BUN* blood urea nitrogen, *FENa* fractional excretion of sodium; **P < 0.01 vs. control; ##*P* < 0.01 vs. LPS, *n* = 10 in each group

**Fig. 2:** Diacerein ameliorated kidney injury in endotoxemic mice. **a** and **b** Mice were injected intraperitoneally with lipopolysaccharide (LPS, 10 mg/kg) for 24 h, and then treated with diacerein (15 mg/kg/day) for a further 48 h. Histological analysis of representative renal cortex (**a**) and medulla (**b**) slides of control, LPS, LPS + DMSO and LPS + Diacerein groups. *n* = 8 in each group (magnification, 100×). Arrows indicate pathologic changes, such as glomerular congestion and atrophy, interstitial hemorrhages, and epithelial cell necrosis and shedding in cortex, and erythrocyte extravasation, cast formation, tubular collapse and collecting duct necrosis in medulla. Diacerein treatment attenuated renal damage induced by endotoxemia

### Diacerein inhibited inflammatory response in kidney of endotoxemic mice

We next determined the effects of diacerein on the inflammatory response induced by LPS. Results of ELISA revealed that LPS significantly increased IL-1β, TNF-α, MCP-1 and NOS-2 levels in kidney tissues. However, diacerein treatment markedly inhibited the increased levels of these inflammatory cytokines (Fig. 3a-d). Notably, immunohistochemical staining of F4/80 expression showed that diacerein markedly inhibited macrophage infiltration in kidney tissues, as evident by a 54% reduction compared with LPS-treated mice alone (Fig. 3e and f).

**Fig. 3:** Diacerein protected against LPS-induced inflammatory response of renal tissue. **a**-**d** After the 72-h experimental period, the whole kidneys of each group were harvested. Levels of interleukin-1β (IL-1β) (**a**), tumor necrosis factor-α (TNF-α) (**b**), monocyte chemoattractant protein-1 (MCP-1) (**c**) and nitric oxide synthase 2 (NOS-2) (**d**) determined by ELISA were inhibited after diacerein treatment. **e** Immunohistochemical staining of F4/80 in the kidneys isolated from each group (magnification, 100×) (arrows). **f** Quantitation of F4/80 was determined by computer-based morphometric analysis, which showed that diacerein markedly inhibited infiltration of macrophages in kidney tissues **P < 0.01 vs. control, ##*P* < 0.01 vs. LPS, *n* = 6 in each group

### Diacerein prevented downregulation of renal AQPs in mice with endotoxemic AKI

Figure 4 shows the effects of diacerein on renal AQP expression. Mice after LPS administration demonstrated significantly decreased AQP1 expression compared with control mice. However, diacerein treatment blocked the reduction of AQP1. The expression of AQP1 was approximately 2.5-fold higher than in mice treated with LPS alone (Fig. 4a). Consistently, the decrease of AQP2 and AQP3 expression in LPS-treated mice was also significantly prevented by diacerein. The expression of AQP2 and AQP3 was approximately 4-fold and 2-fold higher than in untreated endotoxemic mice, respectively (Fig. 4b and c).

**Fig. 4:** Diacerein attenuated downregulation of renal AQP expression in endotoxemic mice. **a**-**c** Protein expression of aquaporin 1 (AQP1) (**a**), AQP2 (**b**) and AQP3 (**c**) in kidney was determined by western blotting. Diacerein significantly inhibited lipopolysaccharide (LPS)-induced decrease of AQP1, AQP2 and AQP3 expression. **P < 0.01 vs. control, ##*P* < 0.01 vs. LPS, *n* = 6 in each group

### Diacerein attenuated endotoxemia-induced downregulation of sodium transporters

As shown in Fig. 5a, renal Na,K-ATPase α1 expression was significantly decreased in LPS-treated mice compared with control mice. In contrast, diacerein treatment prevented the reduction of Na,K-ATPase α1 expression. Furthermore, LPS insult also showed decreased expression of NHE3 compared with control mice. However, diacerein treatment almost completely restored the NHE3 expression to the level of control mice (Fig. 5b). Similar to the changes of Na,K-ATPase α1 and NHE3 expression, the reduced NKCC2 expression was significantly inhibited by diacerein treatment (Fig. 5c).

**Fig. 5:** Diacerein prevented downregulation of renal sodium transporter expression in endotoxemic mice. **a**-**c** Western blotting analysis of Na,K-ATPase α1 (**a**), apical type 3 Na/H exchanger (NHE3) (**b**) and Na-K-2Cl cotransporter (NKCC2) (**c**) in renal tissues of each group. Downregulation of renal sodium transporter expression in endotoxemic mice was markedly reversed by diacerein treatment. **P < 0.01 vs. control, ##*P* < 0.01 vs. LPS, *n* = 6 in each group

### Diacerein prevented the LPS-induced inflammatory response and decrease of AQP and sodium transporter expression in HK-2 cells

To confirm the in vivo findings reported above, HK-2 cells exposed to LPS were concurrently exposed to diacerein or IL-1β siRNA. Expectedly, IL-1β, TNF-α, MCP-1 and NOS-2 levels were increased in LPS-treated HK-2 cells and this increase was attenuated by diacerein or IL-1β siRNA treatment (Fig. 6a-d). Moreover, western blotting showed that LPS also dramatically decreased protein expression of AQP1, AQP2, AQP3, Na,K-ATPase α1, NHE3 and NKCC2 in HK-2 cells. However, these changes of AQP and sodium transporter expression were blocked by diacerein or IL-1β siRNA treatment (Fig. 6e-j).

**Fig. 6:** Effects of diacerein and IL-1β inhibition on AQP and sodium transporter expression after LPS treatment in HK-2 cells. **a-d** The cells were pretreated with diacerein (1 μM) for 1 h, interleukin-1β (IL-1β) siRNA (Si- IL-1β), or negative siRNA (NS) for 48 h before lipopolysaccharide (LPS, 1 μg/mL) incubation for a further 48 h. Levels of IL-1β (**a**), tumor necrosis factor-α (TNF-α) (**b**), monocyte chemoattractant protein-1 (MCP-1) (**c**) and nitric oxide synthase 2 (NOS-2) (**d**) induced by LPS were inhibited by diacerein or IL-1β siRNA treatment. **e**-**j** Protein expression of aquaporin 1 (AQP1) (**e**), AQP2 (**f**), AQP (**g**), Na,K-ATPase α1 (**h**), apical type 3 Na/H exchanger (NHE3) (**i**) and Na-K-2Cl cotransporter (NKCC2) (**j**) was examined by western blotting. LPS-induced decreases of AQP and sodium transporter expression were attenuated by diacerein or IL-1β siRNA treatment. **P < 0.01 vs. control, ##*P* < 0.01 vs. LPS, *n* = 6

## Discussion

In the present study, we provide evidence that diacerein improves renal function in association with histopathological changes and alleviates renal inflammation in mice with endotoxemic AKI. Additionally, diacerein or IL-1β knockdown inhibits the LPS-induced decrease of AQP and sodium transporter expression. The highlight of our work is that diacerein not only attenuates renal inflammation but also alters tubular water and sodium handing, leading to an improvement of renal function.

AKI is characterized by a severe reduction in glomerular filtration rate and decline in renal function as measured by urine output, creatinine, BUN as well as urine osmolarity [20]. Here, our data revealed that the renal function in endotoxemic AKI mice was significantly impaired. However, diacerein treatment improved renal function, including normalization of the decreased urine volume and osmolarity and the increased creatinine, BUN, FENa and serum osmolarity. Furthermore, diacerein treatment also improved histopathological changes in endotoxemic AKI mice. It has been suggested that the elevation of plasma creatinine is associated with the degree of injury of renal medullary thick ascending limbs [21]. Indeed, we observed obvious medulla damage such as vascular congestion, necrosis of thick ascending limbs, cast formation and debris accumulation in endotoxemic mice. Severe injury was also found in the cortex, such as glomerular damage, vacuole formation and interstitial hemorrhages. However, diacerein administration significantly prevented these morphological injuries.

It has been demonstrated that diacerein suppresses inflammation by inhibiting IL-1β synthesis, accompanied by attenuation of inflammatory cytokine production [17]. More importantly, diacerein has also been shown to improve renal function, in parallel with the reduced inflammation, in diabetic nephropathy in mice as well as doxorubicin nephrotoxicity in obese insulin-resistant rats [18, 19, 22]. Consistent with these studies, we found that diacerein treatment clearly decreased renal inflammatory cytokine secretion as well as macrophage infiltration, in mice with endotoxemic AKI.

Abnormal expression of AQPs is closely associated with the pathophysiology of water balance disorder [2, 23]. AQP1 is highly expressed in the descending thin limb and proximal tubule [5]. Wang et al. showed that AQP1 knockout mice had enhanced tubular injury and aggravated endotoxemia-induced AKI [4]. AQP2 and AQP3 are expressed in collecting duct principal cells and are thought to mediate water transport and reabsorption [24, 25]. Additionally, proximal tubule reabsorption of filtered sodium is also severely compromised during AKI [23]. The decreased expression of sodium transporters, such as Na,K-ATPase, NHE3 and NKCC2, may account for the impairment of tubular sodium reabsorption in AKI [4, 9, 23]. A previous study reported that endotoxemia-induced inflammation led to a marked reduction in AQP expression [2, 26]. An early decrease of AQP2 and sodium transporters has been observed in kidneys of rodents undergoing endotoxemia, accompanied by increased macrophage infiltration and NOS2 expression [27–29]. These studies indicate the critical role of inflammation in water reabsorption and urine concentration. Although diacerein has been shown to ameliorate renal injury in several animal models [18, 19, 22], we are the first to outline a potential mechanism showing that the beneficial effects of diacerein may be associated with the restoration of expression of AQPs and major sodium transporters. Our data revealed that diacerein dramatically attenuated the decrease of AQP1, AQP2, AQP3, Na,K-ATPase α1, NHE3 and NKCC2 expression in endotoxemic AKI mice. Furthermore, in our in vivo study, we found that diacerein treatment or IL-1β inhibition significantly inhibited LPS-induced secretion of inflammatory cytokines and the decrease of AQP and sodium transporter expression.

A clear limitation of the current study is that it is impossible to exactly clarify the potential targets of diacerein. Diacerein is primarily designed as an IL-1β inhibitor, which has been widely used for osteoarthritis treatment by suppressing cartilage degradation synovitis and promoting cartilage synthesis [14]. It is worth noting that several studies have demonstrated a potential anti-inflammatory effect of diacerein by its ability to inhibit synthesis and activity of other pro-inflammatory cytokines, such as TNF-α and IL-6 [16]. Moreover, diacerein also inhibits IκB-α degradation, leading to decreased NF-κB translocation to the nucleus and subsequently reduced nitric oxide and IL-6 production [17]. Importantly, NF-κB regulates AQP2 transcriptional activity and inhibition of NF-κB ameliorates sepsis-induced downregulation of AQP2 [30, 31]. Therefore, in this study, we cannot conclude whether the potentially protective effect of diacerein against renal inflammation and injury is due to inhibition of IL-1β. Further studies are needed to illustrate the mechanisms underlying the beneficial effects of diacerein on renal function.

In summary, the results of this study clearly demonstrate that diacerein significantly ameliorates endotoxemia-induced AKI by attenuating inflammation and restoring AQP and sodium transporter expression, resulting in improvement of renal function. Our findings suggest that diacerein may represent a viable option for the treatment of endotoxemic AKI.

## Abbreviations

AKI: acute kidney injury
AQP: aquaporin
BUN: blood urea nitrogen
FENa: fractional excretion of sodium
IL-1β: interleukin-1β
LPS: lipopolysaccharide
MCP-1: monocyte chemoattractant protein
NHE3: apical type 3 Na/H exchanger
NKCC2: Na-K-2Cl cotransporter
NOS-2: nitric oxide synthase 2
TNF-α: tumor necrosis factor
